The article "The Influence Mechanism of Information Interaction on Value Cocreation Based on the Smart Healthcare Context" was retracted in 2023. Reasons: unreliable results or conclusions; concerns about the data; concerns about the peer review; concerns about the citations.

# The Influence Mechanism of Information Interaction on Value Cocreation Based on the Smart Healthcare Context

**DOI:** 10.1155/2021/8778092

**Published:** 2021-08-27

**Authors:** Lan Zhang, Xiu Yang, Yuan Zhou, Jialu Sun, Zixiang Lin

**Affiliations:** ^1^School of Accounting, Jilin University of Finance and Economics, Changchun 130017, Jilin, China; ^2^Accounting&Auditing College, Guangxi University of Finance and Economics, Nanning 530003, Guangxi, China

## Abstract

In recent years, the Chinese government has issued a series of deepening reform policies around smart healthcare, established a diversified technical basis and environmental protection, and deeply excavated the derivative value of healthcare information, aiming to provide high-quality healthcare services for patients. Information interaction in the context of smart healthcare is a kind of health information interaction completed by users with smart healthcare applications as the hub. It is an application form of social behavior and has an impact on value cocreation. Based on the theory of information interaction and value cocreation, this paper systematically reviews the research on information interaction and value cocreation in the smart healthcare context, analyzes the information interaction mode and information interaction mechanism in the smart healthcare context, constructs a theoretical model of the impact of information interaction on value cocreation, and empirically tests the relationship between information interaction and value cocreation in the smart healthcare context. The research of this paper aims to provide high-quality information interaction services for smart healthcare users, promote the dimensional management of information behavior in the context of smart healthcare, and promote the continuous improvement of the operation and management of smart healthcare.

## 1. Introduction

With the rapid development of Internet of Things, big data, artificial intelligence, and other technologies, emerging applications and service models have gradually penetrated into all aspects of the medical and health field. So far, the informatization development process of the medical industry has entered the stage of smart healthcare. Medical institutions have rapidly promoted intelligent convenience measures such as online consultation, follow-up evaluation, and AI diagnosis. With the improvement of the recognition of the majority of patients and doctors on the application experience of smart healthcare, it has become an important issue for medical and health departments and institutions to deeply understand the internal mechanism of information interaction to ensure the continuous, smooth, and healthy development of information interaction and alleviate the imbalance between medical demand and medical resource supply. In the new generation of the information technology environment, information interaction is a new core ability. Smart healthcare provides an efficient diagnosis and treatment environment for doctors and patients. Research on information interaction behavior in the context of smart healthcare can further tap the needs of users, so as to improve the efficiency of health management [1].

Most of the previous studies are based on the intelligent transformation of objective medical services and do not integrate the interaction between users and its impact on value cocreation into the smart healthcare service model. In fact, interaction has been throughout the development of value cocreation theory, and it is an important way of value cocreation [2]. Interaction is also an important driver of value creation [3, 4]. Based on the perspective of information interaction, this paper unlocks the connotation and composition of the smart healthcare context, explores the mode and mechanism of information interaction in the smart healthcare context, and empirically studies the impact of information interaction on value cocreation in the smart healthcare context. The main research contents are as follows: firstly, explore the basic content of information interaction in the context of smart healthcare by combining the mode and the mechanism of information interaction in the context of smart healthcare; secondly, through the analysis of the impact of information interaction, to explore the impact of user participation value cocreation on both doctors and patients to understand the role. Following the SPS (structured-pragmatic-situational) case study method [5], data collection, screening, and verification are carried out to ensure the calibration of the theory, data, and model. The theoretical analysis framework is constantly used to guide data collection and to improve the theoretical analysis framework with data. Thirdly, this paper conducts an empirical study on the information interaction of patient users in the context of smart healthcare and its impact on value cocreation from the perspective of user behavior, so as to provide basis and suggestions for the research, management, and development of related theories of smart healthcare.

The possible contributions of this paper are mainly reflected in three aspects. First, information interaction is the most direct way for people to acquire knowledge. Using this information interaction can promote the interest expression of information users and meet the needs of information users. Second, it can deepen the application of value cocreation theory in the healthcare field. Medical treatment is a field requiring high participation of both doctors and patients. The effect of diagnosis and treatment of diseases depends largely on the degree of active participation of patients. Third, it provides selection and decision-making basis for smart healthcare users. This paper analyzes the value cocreation brought by the interaction mode in the context of smart healthcare and actively explores the value cocreation brought by the integration of the internet and the medical industry.

## 2. Theory

### 2.1. Information Interaction in the Context of Smart Healthcare

Jamil et al. [6] proposed that smart healthcare can create a smart healthcare drug system with a drug supply chain on the blockchain to conduct drug record transactions to solve the problem of counterfeit and shoddy drugs entering the market. Based on the introduction of Saudi Arabia's smart healthcare system, HajAli et al. [7] believed that it can make appointments, update data, and extract medical records by collecting patients' digital ID cards or fingerprints, so as to realize the data sharing of hospital information, medical centers, and patients' medical records. With the help of intelligent technology, smart healthcare can deeply perceive user situations, fully tap user needs, and seamlessly embed it into users' diagnosis and treatment, scientific research, and learning activities to provide a large number of rich, efficient, and accurate smart healthcare services. Therefore, in this paper, smart healthcare context is defined as a diagnosis and treatment process that causes positive emotional response and stimulates behavioral potential on users with the help of technologies such as the Internet of Things, big data, and artificial intelligence in the process of medical activities. It takes the life cycle as the guide, the user needs as the center, the information behavior as the link, and the individual data as the support to enhance the understanding of the real intention of users in the context of smart healthcare treatment, so as to improve the information relevance and user satisfaction.

According to Moggridge, this paper defines information interaction behavior as the behavior that two or more cognitive subjects transmit, communicate, and share information with each other by means of a certain communication medium. Information interaction in the context of smart healthcare refers to the transmission and exchange of medical knowledge through continuous sending and receiving of information between patients and doctors, systems, and devices. Each link in the process of information interaction affects and interacts with each other to provide users with accurate and perfect information services. Kim [8] pointed out that, in the smart healthcare system, many medical devices are distributed in hot areas such as stations and medical centers, and such high-density distribution of medical devices will lead to a serious decline in the communication performance. Based on this, a distributed coexistence mitigation scheme for the smart healthcare system based on the Internet of Things was proposed, which can dynamically avoid interference in the coexistence environment and ensure the reliability of medical communication. The extensive construction of the Internet of Things in the information interaction environment can be applied in medical emergency. In the aspect of physical sign monitoring, the sensor can continuously measure the user's physiological parameters for a long time so that the doctor can grasp the patient's physical sign status in time. Therefore, the Internet of Things has become the best way to build an interactive environment of medical information, so as to comprehensively understand the behavioral intention of smart healthcare users in different situations such as medical institutions, telemedicine, and homecare and provide personalized services.

### 2.2. Value Cocreation

Ramirez [9] first coined the term value cocreation, describing it as a “galaxy of values.” Prahalad and Ramaswamy [10] put the concept into a hot spot by studying value cocreation based on consumer experience. Then, Prahalad and Ramaswamy [11] proposed the theory of value cocreation from the perspective of strategic management. The two scholars' core views on value cocreation can be summarized into three points: ① interactive creation of value and the interaction quality between enterprises and users directly affect whether enterprises can provide unique experience environment for users. ② Dialogue, access, risk management, and transparency (DART) are the four basic elements of value cocreation, and personalized and high-quality user experience is the core of value cocreation. ③ In order to realize value cocreation, hospitals also need to build new strategic capital and new core capabilities.

Vargo et al. [12] shifted the study of value cocreation from the perspective of service science to the network relationship, emphasizing the interaction within and between service systems. However, both service exchange and value cocreation are affected by social forces in reality. The position and role of suppliers and customers in the social structure all affect the understanding and action of value cocreation [13], and value creation occurs in a more complex situation. Based on the expansion of service-led logic, the perspective of the service ecosystem has become an important research perspective to study value cocreation in the current complex network environment. After Vargo and Lusch [14] proposed the concept, scholars began to conduct in-depth research on relevant theories [15–20]. In recent years, with the transformation of the value creation system and the change of the role and status of users, scholars have realized the importance of value cocreation. No matter it is an enterprise or a public institution hospital, value cocreation must be valued in order to gain competitive advantage in the future [21, 22]. MC Coll-Kennedy [23, 24] proposed patient value cocreation, which refers to the benefits realized by patients and medical service providers through multiparty interaction and resource integration in the service network. The two are resource integrators. Operational resources (such as knowledge and skills) and objective resources (such as equipment, drugs, and financial resources) are integrated to achieve common benefits.

### 2.3. The Relationship between Information Interaction and Value Cocreation in the Context of Smart Healthcare

In the context of smart healthcare, the existing resources can be fully utilized to alleviate the pressure of the population, economy, and technology, adjust the contradiction between supply and demand, and enhance the connection between patients and medical personnel. Through the effective interaction between the two, practical problems caused by the traditional medical model can be alleviated. Information interaction is valuable, scarce, and difficult to be imitated and used by organizations. It is an overall and strategic enterprise core competence. In terms of empirical research, many scholars regard interaction-related activities, interaction frequency and content, and effective modern communication ability with patients as the influencing factors of value cocreation. The results show that the above factors have a significant positive impact on value cocreation, and interaction is an important driving force of value creation ([22, 25–28], etc.). Prahalad and Ramaswamy [11] believed that the value cocreation process is an interactive process. By managing the interaction of information among patients, doctors, and hospitals, value co-creation is created. For example, doctors and patients make concerted efforts to improve the matching degree of medical service supply and demand by means of extensive information exchange, which will contribute to the effect of disease diagnosis and treatment, improve medical quality, and ultimately enhance value.

Information interaction is an important means to realize value cocreation, and value cocreation is the starting point of building information interaction ability and the standard of measuring the effectiveness and quality of information interaction ability, which runs through the whole process of building and applying information interaction ability. Both complement each other and have inherent consistency. Lan et al. [29] found that users with high responsibility perception are more willing to adopt value cocreation behavior through interviews and questionnaires. Luu [30] found that CSR was positively correlated with the enthusiasm of customers to participate in value cocreation through a questionnaire survey. Vazquez-Casielles et al. [31] found that customers who participated in cocreation had a higher sense of satisfaction and shopping pleasure than those who did not participate and were willing to spread a good reputation for suppliers. It can be seen that interaction is an important strategy to promote value cocreation, which has been a general consensus and has an important role to promote the medical industry which has been a big step towards the wisdom, network, and technology.

## 3. Exploratory Case Analysis

### 3.1. Research Design

#### 3.1.1. Method Selection

Eisenhardt [32] argued that case study is considered to be very effective when a study begins with little knowledge of the issues raised or attempts to enter a research issue from a new perspective. Information interaction proposed in this study is a new perspective, and academic research on information interaction and its framework is still in its infancy. On the contrary, this paper explores the impact of information interaction on value cocreation. Yin [33] believed that the exploratory case study method is particularly suitable for solving the above problems. This paper follows the SPS (structured-pragmatic-situational) case study methodology [5].

#### 3.1.2. Case Selection

The development of the smart healthcare service system needs to be oriented towards patients, healthcare professionals, medical institutions, and health regulatory and supervisory agencies. The business model of the smart healthcare service platform aims to promote the transformation of traditional relationships in healthcare service systems with the development and application of information technology and form a healthy ecosystem through the industrial aggregation function of the smart healthcare information service platform. The smart healthcare ecosystem, which is formed via multidisciplinary and cross-industry integration, involves many stakeholders, including consumers, policy makers, and regulators, technology providers, service providers, medical service payers, and capital investors. This case study aims to investigate the potential participants of the smart healthcare service platform and understand their needs and value proposition, improve the ability of the platform model to meet the needs of stakeholders, and enhance value cocreation. Accordingly, eight institutions in the developed coastal areas of South China, including two hospitals and six stakeholders, were selected for the survey in this study. To ensure the reliability of the information in the case study, the availability of information and the industrial characteristics and representativeness of the institutions were considered when selecting the interview samples.

#### 3.1.3. Data Collection

To ensure that the design of the platform business model was reasonable, the stakeholders of the smart healthcare information service platform were interviewed. For the institutions interviewed, we collected first-hand data through field research and semistructured interviews, and after the interviews, we verified and supplemented the data through online channels such as emails and phone calls. In addition, second-hand data were obtained for quantitative analysis and verification. The data sources for the stakeholders in this case study are shown in Table 1.

### 3.2. Case Description

Through the systematic analysis of the data of the primary and second-hand data, it is found that the process of information interaction in the context of smart healthcare is a dynamic development and continuous updating process. Each component element is interrelated and affects each other. In the context of smart healthcare, from inquiry, examination, surgery, and nursing to rehabilitation, all processes of user medical treatment can be recorded, quantified, and perceived. The overall deconstruction of the smart healthcare situation takes user needs as the breakthrough point, combines the medical treatment process and doctor-patient interaction, and promotes the flow of healthcare information and further realizes the value-added information through the interaction between user subjects. Smart healthcare context includes not only simple and intuitive environment and system situation, such as geographical location and system parameters, but also users' own cognition, behavior, emotion, and other deep situations. Based on the research on the connotation and characteristics of the smart healthcare context, this paper divides the smart healthcare context into smart hospital situation, regional health situation, and family doctor situation.

Information interaction in the smart healthcare context refers to the continuous sending and receiving of information between patients and doctors, systems, and equipment, so as to realize the transmission and exchange of medical knowledge. Information interaction is divided into two modes: one-way interaction and two-way interaction. One-way interaction means that the attributes between the sender and the receiver are unchanged. One side only sends information, and the other side only receives information. In the two-way interaction, the attributes between the sender and the receiver are constantly exchanged, and the subjects of both sides are both information senders and information receivers. In the process of two-way interaction, medical information generates medical knowledge in the continuous accumulation. The information exchange in the context of smart healthcare can establish the knowledge expression and communication between the subjects and then assist the diagnosis and treatment process to improve the quality of health management.

### 3.3. Case Analysis

The analysis of the smart healthcare context is the basis of information interaction research in the smart healthcare context. The characteristics are the premise of understanding and studying user information interaction. The process of information interaction under the interaction of the smart healthcare context is a dynamically developed, continuously updated process, and every component affects each other, which in turn constitutes an organic overall that uses the user-centered and promotes information flow.

#### 3.3.1. Information Interaction Mode in the Smart Healthcare Context

Man-machine interaction mode, machine-machine interaction mode, and man-man interaction mode are three basic modes of information interaction. Man-machine interaction mode is the most basic information interaction mode. Machine-machine interaction mode is the core information interactive mode. Man-man interaction mode is the ultimate goal of information interaction under the smart healthcare context. In the smart healthcare context, man-man interaction is the premise and basis for the man-machine interaction mode and machine-machine interaction mode. The process of building interactive modes under smart healthcare contexts is to explore how to achieve man-man interaction through man-machine interaction and machine-machine interaction. Therefore, in the smart healthcare information interaction mode, the three information interaction modes are not born at the same time, but have a progressive relationship. Medical data are always the center of the information interaction process. It is used to observe the flow of medical data. The operation process of the information interaction mode in the smart healthcare context can be explained below: man-machine interaction realizes the machine's medical data collection. Machine-machine interaction achieves the traffic acquisition data in the smart healthcare system and finally achieves medical data from the machine to the output of the machine, that is, the information interaction. In this way, the circulation of medical data in the smart healthcare system is realized.

#### 3.3.2. Information Interaction Mechanism in the Smart Healthcare Context

The information interaction in the smart healthcare context is not a static unidirectional process, but a dynamic two-way development process, consisting of six elements of information senders, coding, media, information recipients, decoding, and feedback. The information interaction in the intelligence situation can be roughly divided into four stages: information release stage, information transmission stage, information acquisition stage, and information feedback stage. The operation of information interaction in the smart healthcare context is relatively complex, which is a diversified concept with a very large coverage. In addition to the simple model process construction, it also involves the interaction between users, medical staff, medical institutions, and other subjects.  Figure 1 reveals the information interaction mechanism in the smart healthcare context. It mainly solves the problems in three aspects. First, analyze the connection between various users, collect the main information, and fully utilize information resources. Second, the information interaction relationship in smart healthcare context should be properly handled based on the actual needs of the user, combined with the construction of the online platform, ensuring that man-machine interaction needs to be effectively satisfied. Third, use large data to assist medical decisions, support management applications, enrich research databases, etc., and achieve cross-regional information sharing.

From the actual situation, the main purpose of the information interaction in the interactive situation in the intelligence situation is to display the entire process of user collection information based on the information interaction between man-machine-man, combined with the application of large data technology, analyzing the patient's direct impact, understand its true state feedback, and complete the interaction between users with a scientific reasonable approach. User's physiological and safety needs, as well as respect and self-actualization needs, drive the generation of their health expectation, psychological expression, and other motivations. When the internal needs and external incentives reach a certain point of eruption, users will be motivated to generate information interaction. The user has willingness to interact with medical information, and there is an act of information release, information transmission, information acquisition, and information feedback. The development of information interaction relies on user networks, equipment networks, and information networks formed between the subjects, and under stable and orderly network structures, information interaction can be used to play its maximum performance.

### 3.4. The Relationship between Information Interaction and Value Cocreation in the Context of Smart Healthcare

At the beginning of value cocreation research, interaction was recognized as the basic analysis unit of value cocreation; that is, value cocreation is interactive. Interaction has been running through the development of value cocreation theory, and it is the basis, important place, and important way of value cocreation [11], which is a better choice for organizations to achieve value [34]. Prahalad and Ramaswamy argued that the value cocreation process is an interaction process.

The information interaction under the context of smart healthcare is not for the information interaction of research and development, not for marketing management information interaction, and not for supply chain management information interaction, but is more representing information interaction in evolution. Evolving information interaction refers to the enterprise in order to create the user experience, through configuration, application, and integration of a variety of interactive information infrastructures, information interaction of human resources and intangible resources, and information interaction with the user, the user community, and partners such as the core of the value network members jointly built for the future value creation ability, so as to obtain the competitive advantage of information interaction ability. In the smart healthcare context, the information interaction and value-shared relationship framework is shown in Figure 2.

Information interactive resources form information interactive ability through dedicated allocation and application integration and then drive the formation of value cocreation. Information interaction is the important means to realize value creation. Value cocreation is the starting point of constructing information interaction ability and the standard of measuring the effect quality of information interaction, which runs through the whole process of constructing and applying information interaction ability. The two complement each other and have internal consistency. It can be seen that interaction is an important strategy to promote value cocreation, which has been a general consensus, and it has an important role to promote the medical industry, which has strikingly moved towards the wisdom, network, and technology.

## 4. Empirical Analysis

### 4.1. Assumption

As can be seen from the above case study, information interaction in the context of smart healthcare is that patients continuously send and receive information between doctors, systems, and devices, so as to realize the transmission and exchange of medical knowledge. In the process of two-way interaction, healthcare information generates healthcare knowledge in the continuous accumulation. Through interaction and effective integration, all kinds of knowledge are finally applied to the treatment plan of patients. In this process, the value of information exchange is reflected. From the user's perspective, the information interaction among users, medical institutions, and value network members is the key factor that determines the quality of user experience jointly created. The interaction between medical institutions and value network members can understand user needs from more channels and, at the same time, can ensure the rapid response to medical institutions, so as to improve the quality of user experience, and cocreation of user experience is the purpose of value cocreation. Therefore, it can be said that the stronger the information exchange ability of medical institutions, the more unique and high-quality user experience they will be able to create, so as to achieve value cocreation. Payne et al. [35] believed that interaction is the basis of value cocreation, value cocreation cannot be realized without interaction, and interactive ability has become a new driving force for value cocreation.

In addition, the source of value for medical institutions in the context of smart healthcare increasingly relies on the cocreation of experiences. So medical institutions must enhance the ability of information interaction and build a robust user experience environment to further promote the co-creation of experience. According to Prahalad and Ramaswamy [11], value cocreation is formed by the heterogeneous interaction between users and medical institutions at each node of the value network, and it is an important strategy to promote value cocreation to improve the interaction quality between medical institutions, users, and partners and provide users with a unique experience environment. Therefore, medical institutions must enhance the ability of information interaction to create personalized experience for users and sequentially achieve value cocreation. As a result, based on the above analysis, this paper proposes the following hypotheses:

  H1: information interaction can promote value cocreation in the context of smart healthcare

### 4.2. Variable Measure

In the discussion of the empirical analysis of this paper, the variables that need to be determined are those related to information interaction (explanatory variable) and those related indicators that reflect the level of value cocreation (explained variable).

#### 4.2.1. Information Interaction Willingness (*X*1)

Information interaction behavior is the user's action driven by the willingness, and its generation process has experienced from motivation to execution. Based on the ideas of previous scholars, Wang Xiwei and others in the use of live web app behavior study found that, after the live webcast experience, users usually cannot be with the ‘cutoff contact' host, but will watch the corresponding live or turn to other network platforms, and continue to focus on the host's Weibo and WeChat. If users have a strong willingness to use smart healthcare under the joint action of information, technology, environment, and other factors, they will be driven to actively generate information interaction. The information interaction willingness measure items are shown in Table 2.

#### 4.2.2. Information Interaction Behavior (*X*2)

Information interaction behavior refers to a series of actions made by two or more parties after reaching the intention of information interaction, including information exchange, information extraction, data analysis, and data feedback. Through the information interaction behavior, the information releasing party and the receiving party obtain the information they need or the potential benefits. The information interaction behavior measure items are shown in Table 3.

#### 4.2.3. Information Interaction Ability (*X*3)

This paper studies the subjects related to healthcare and divides them according to the contact mechanism of community members in the process of information interaction. Information interaction between members of online medical communities can be divided into strong and weak, which are vividly called “strong link” and “weak link.” For example, attention relationship is considered to be a relatively stable “strong link,” which limits the effect of information interaction ability of each node. The information interaction ability measure items are shown in Table 4.

#### 4.2.4. Value Cocreation (*Y*)

Value cocreation is a very abstract concept. Scholars reflect value cocreation through measuring value cocreation activities, so as to achieve the purpose of measuring value cocreation. Based on the DART model and combining the characteristics of the medical industry, this paper designs the initial scale of value cocreation in the smart medical industry by consulting experts and discussing with the coordination group. The value cocreation measure items are shown in Table 5.

### 4.3. Data Collection and Sample Characteristics

In the context of smart healthcare, the Internet of Things has been comprehensively applied in the healthcare field. It includes health education, medical information inquiry, electronic health records, disease risk assessment, online disease consultation, electronic prescription, remote consultation, remote treatment, and rehabilitation and other forms of health and medical services. Specifically, patients can make correct health management through their own health data and health intervention. Doctors can continue to learn from medical data and realize auxiliary diagnosis. Drug companies can use treatment data for drug research and development and precision marketing. Insurance companies can make reasonable premium pricing based on coverage and treatment data and prevent overtreatment. From the perspective of time, doctors can make use of their idle time to conduct online diagnosis and treatment. In space, doctors can carry out remote consultation, remote therapy, and so on.

This paper holds that internet medicine is an expression of the in-depth application of smart healthcare context information interaction. Therefore, 22 typical listed internet medical companies in the context of smart healthcare were selected, combined with the status and scale of the listed companies and the financial data of the input-output of smart healthcare projects. The explanatory and explained variables were scored on a 10-point scale: score 5 is divided into basic, higher than the base score, and decrease lower than the base score; score with a point value between 1 and 10 is free distribution. Through the analysis of the relevant financial data and business investment activities of the 22 listed internet medical companies with different market segments, the samples are firstly sorted according to the overall application level of smart healthcare services, considering only the activities of information interaction part and the value created thereby (value cocreation). Then, the index of a sample company whose development level is in the middle is determined as the measurement standard. Finally, the score of the influence of information interaction on value co-creation of the 22 Internet medical enterprises was obtained through comparative analysis with the measurement standard company (rank them from lowest to highest), shown in Table 6.

### 4.4. Data Analysis and Hypothesis Testing

#### 4.4.1. Data Export

Relevant data were imported into the EViews model for correlation test in order to verify the influence of information interaction on value cocreation in the context of smart healthcare. The results are shown in Table 7.

#### 4.4.2. Feasibility Test of the Data

**Step 1 .**

*R*^2^ test.

From the experimental data, it can be seen that *R*^2^ = 0.986739 and adjusted *R*^2^ = 0.984529. The closer this statistic is to 1, the higher the fitting degree of the model will be. Therefore, this model meets the *R*^2^ test.

**Step 2 .**

The *T*-test.

According to the data in the table and the lookup table, the critical value of *T* is 1.734 (significance level *α* = 0.05). The degree of freedom is 18, and the explanatory variable's *T* value is *X*1 = 3.825414, *X*2 = 4.513978, and *X*3 = 5.5413978, respectively. It can be seen that the *T* value is all greater than the critical value, satisfying the *T*-test, which rejects the null hypothesis.

**Step 3 .**

The *F*-test.

*F* of the experimental results is 446.4534. When the degree of freedom is (3, 18) and the significance level is *α* = 0.05, *Fα* = 3.16 and *F* > *Fα* meet the *F*-test and reject the null hypothesis, and the *t*-test is consistent with the *F*-test.

#### 4.4.3. Empirical Conclusion

In summary, the empirical conclusion is established. Information interaction has a significant positive impact on value cocreation in the context of smart healthcare.

## 5. Conclusion and Suggestion

It can be seen from the above empirical analysis results that information interaction has an impact on value cocreation and presents a positive correlation trend. That is, in the context of smart healthcare treatment, the stronger the information interaction ability is, the greater the value cocreation will be. It is an inevitable trend to introduce scientific and technological innovations in the process of medical development. Research on information interaction behavior in the context of smart healthcare can enhance the connection between patients and medical staff and alleviate the practical problems caused by the traditional medical model through the effective interaction between the two. Information interaction is one of the most direct ways for people to acquire knowledge. Promoting the communication and interaction between users can promote the expression of interests of information users and meet the connotation needs of information users.

In terms of theory, firstly, this study obtains the connotation of value cocreation behavior in the smart healthcare industry based on the DART model, which laid a theoretical foundation for the development of the scale and subsequent empirical research. Secondly, on the basis of the literature review, reference to relevant domestic and foreign survey scales and questionnaires, and coordination of group discussion, a value cocreation behavior scale based on the DART model is developed to lay a foundation for the quantitative measurement of value cocreation behavior. Finally, the influencing factors of value cocreation behavior were found, and corresponding countermeasures were put forward to improve the enthusiasm of patients to participate in value cocreation. The analysis shows that self-efficacy, responsibility cognition, and perceived value cocreation of doctors have positive effects on value cocreation behavior.

Smart healthcare is regarded as a strategic tool to realize the people-oriented integrated service model. The smart healthcare context presented in this paper is based on the framework of smart healthcare proposed by the World Health Organization (WHO). The problems faced by the development of smart healthcare in China were analyzed, and the possible policy paths to improve the development of smart healthcare in China were proposed, which were also applicable to other countries. Therefore, in order to optimize the interaction effect of smart healthcare treatment, the following suggestions are put forward in this paper. The first is to establish a long-term guarantee mechanism for the operation of smart healthcare treatment. To build the operation management team, the current medical information service is still in the content-oriented stage, rather than the user demand-oriented stage, which affects the user medical information interaction effect to a certain extent. The second is to establish a friendly information exchange network environment. It is necessary to pay attention to the cultivation of smart healthcare talents, pay attention to the skill training and professional accomplishment improvement of practitioners, and ensure that every employee can be skilled in operating service skills and has a certain understanding of the relevant network platform and information technology knowledge. The third is to innovate on the information interaction service mode. On the basis of the existing information interaction service mode, constantly introduce the concept that can promote the realization of information interaction to improve the smart healthcare service. It is necessary to establish and improve the communication mechanism between medical staff and patients, which is helpful for medical staff to conveniently, timely, and accurately grasp the needs of patients and realize the improvement of service quality through good interaction between the two sides.

## Figures and Tables

**Figure 1:** Information interaction model in the context of smart healthcare treatment.

**Figure 2:** Theoretical framework diagram of information interaction and value cocreation in the context of smart healthcare.

**Table 1:** Data sources for the case study.

Type of institution	Interviewee	Type of interview	Field observation	Second-hand data
Policy makers and regulators	WM Health Administration	One field interview with a person in charge of the relevant department	Field visit to the relevant department	Government web page data and related news reports

Medical institutions	People's Hospital of WM	Field interviews with three people in charge of relevant departments, several communications via phone calls and social media	Field inspection of the implementation of medical informatization and management of the information service platform	Official website, related reports, and internal information
	WM Heath Service Center	One field interview with a person in charge of the relevant department	Field inspection of the degree of network informatization	Official website, related reports, and internal information

Research and development (R&D) institutions	R&D Center, School of Pharmacy, XJ University	One field interview with a person in charge	Field visits to research centers and laboratories	Research achievements and news reporting from the institution's official website
	WM United Laboratories	One field interview with a person in charge of the R&D department	Field visits to R&D base, firm headquarters, and exhibition center	News reporting from the institution's official website, industry development reports, and annual reports

Suppliers	WM Medical Service Management Co., Ltd.	One field interview with a marketing manager	Field visit to the business department of the firm	News reporting about the firm and internal information
	WM Pharmaceutical Co., Ltd.	One field interview with a retail store manager	Field visit to the retail store	Firm's internal reports, annual reports, and official website
	HT Medical Equipment Co., Ltd.	One field interview with a marketing manager	Field visit to the firm's headquarters	Firm's internal reports, annual reports, and official website

**Table 2:** Information interaction willingness measure.

Variable name	Measurement items	Coding	Source of theory
Information interaction willingness	I would like to use smart healthcare applications	W1	Venkatesh et al. [36]; Fishbein, Ajzen [37]
	I am willing to pay for smart healthcare applications	W2	
	I would recommend others to use smart healthcare apps	W3	

**Table 3:** Information interaction behavior measure.

Variable name	Measurement items	Coding	Source of theory
Variable measure	I often use smart health apps to get medical information	B1	Venkatesh et al. [36]
	I am an active user of smart healthcare applications	B2	
	I often follow the updates of smart healthcare products and applications	B3	Mark et al. [38]

**Table 4:** Information interaction ability measure.

Variable name	Measurement items	Coding	Source of theory
Information interaction ability	I learned about smart healthcare first-hand from other people	A1	Jiang Kan,etc. [39] Chen Yuan,ect. [40] Cao Xueyan,ect. [41]
	I learned about smart healthcare by filling in a questionnaire offline	A2	
	I have read about smart healthcare on social media	A3	

**Table 5:** Value cocreation measure.

Variable name	Measurement items	Coding	Source of theory
Value cocreated	Users can easily access the smart healthcare information platform to obtain services	V1	Taghizadeh et al. [42] Mazur and Zaborek [43] Prahalad and Ramaswamy [11]
	Smart healthcare platform will actively and effectively solve problems for users	V2	
	Smart healthcare platform will protect users' personal information	V3	

**Table 6:** Rating the impact of information interaction on value cocreation.

Value cocreation (*Y* ∗ 3)		Information interaction willingness (*X*1)	Information interaction behavior (*X*2)	Information interaction ability (*X*3)
A1	10.2	4	3	3
A2	10.8	4	4	3
A3	11.4	4	5	3
A4	12	5	4	4
A5	12.3	4	5	5
A6	14.7	4	5	5
A7	15	5	5	5
A8	15.6	5	6	5
A9	16.8	6	6	5
A10	17.7	6	7	5
A11	17.7	5	7	6
A12	19.8	6	7	6
A13	21	6	7	7
A14	22.8	7	7	7
A15	22.8	6	8	7
A16	24	7	7	9
A17	27.3	7	9	8
A18	27.6	7	9	9
A19	28.5	8	10	9
A20	29.4	9	9	9
A21	29.7	9	10	9
A22	29.7	9	10	9

**Table 7:** Data analysis results.

Dependent variable: *Y*				
Method: least squares				
Date: 06/10/21; time: 00:01				
Sample: 1 22				
Included observations: 22				
Variable	Coefficient	Std. error	*t*-statistic	Prob.
*C*	−2.486653	0.706511	−3.519626	0.0024
*X*1	1.067627	0.279088	3.825414	0.0012
*X*2	1.120217	0.248166	4.513978	0.0003
*X*3	1.315068	0.237363	5.540322	0.0000
*R*-squared	0.986739	Mean dependent var		19.85455
Adjusted *R*-squared	0.984529	SD dependent var		6.772826
SE of regression	0.842426	Akaike information criterion		2.657905
Sum squared resid	12.77428	Schwarz criterion		2.856276
Log likelihood	−25.23695	Hannan–Quinn criter.		2.704635
*F*-statistic	446.4534	Durbin–Watson stat		1.744985
Prob (*F*-statistic)	0.000000					

## Data Availability

The data that support the findings of this study are available from the corresponding author upon reasonable request.

## References

[1] Hui-zi Y., Zhang H.-t., Ma T.-t. (2020). Ect. Research on information interaction behavior and topological structure in the context of smart healthcare treatment. *Journal of Modern Information*.

[2] Prahalad C. K., Ramaswamy V. (2004). Co-creation experiences: the next practice in value creation. *Journal of Interactive Marketing*.

[3] Ballantyne D., Varey R. J. (2006). Creating value-in-use through marketing interaction: the exchange logic of relating, communicating and knowing. *Marketing Theory*.

[4] Tirnea L., Minciu R., Olariu T. R., Dumitrascu V., Neghina A. M., Neghina R. (2014). A rare case of renal hydatidosis in a child with congenital solitary kidney. *Asian Pacific Journal of Tropical Medicine*.

[5] Pan S. L., Tan B. (2011). Demystifying case research: a structured-pragmatic-situational (SPS) approach to conducting case studies. *Information and Organization*.

[6] Jamil F., Hang L., Kim K. H. (2019). A novel medical blockchain model for drug supply chain integrity management in a smart hospital. *Journal of Electronics*.

[7] HajAli F. R. A. (2020). Al-onazi, SKAAL, etc. Using smart card and integrated medical record system (IMRS) for improving health system in Saudi Arabia. *Journal of computer science and network security*.

[8] Kim B. S. (2017). A distributed coexistence mitigation scheme for IOT-based smart healthcare systems. *Journal of information processing systems*.

[9] Ramirez R. (1999). Value Co-production: intellectual origins and implications for practice and research. *Strategic Management Journal*.

[10] Prahalad C. K., Ramaswamy V. (2000). Co-opting customer competence. *Harvard Business Review*.

[11] Prahalad C. K., Ramaswamy V. (2004). Co-creation experiences: the next practice in value creation. *Journal of Interactive Marketing*.

[12] Vargo S. L., Lusch R. F. (2008). Service-dominant logic: continuing the evolution. *Journal of the Academy of Marketing Science*.

[13] Edvardsson B. T. Value co-creation and value-in-context: understanding the influence of duality of structures.

[14] Vargo S. L., Lusch R. F. (2010). From repeat ratronage to value co-creation in service ecosystems: a transcending conceptualization of relationship. *Journal of Business Market Management*.

[15] Vargo S. L., Lusch R. F. (2011). It’s all B2B and beyond: toward a systems perspective of the market. *Industrial Marketing Management*.

[16] Lu S. (2016). *The Effect of Information Interaction Capabilities on Value Co-creation and Competitive Advantage of Firms*.

[17] Chandler J. D., Vargo S. L. (2011). Contextualization and value-in-context: how context frames exchange. *Marketing Theory*.

[18] Lusch R. F., Vargo S. L. (2014). *Service-Dominant Logic: Premises, Perspectives, Possibilities*.

[19] Lusch R. F., Nambisan S. (2015). Service innovation: a service-dominant logic perspective. *MIS Quarterly*.

[20] McColl-Kennedy J. R., Cheung L., Ferrier E. (2015). Co-creating service experience practices. *Journal of Service Management*.

[21] Galvagno M., Dalli D. (2014). Theory of value co-creation: a systematic literature review. *Managing Service Quality*.

[22] Neghina C., Caniels M. C., Bloemer J. M., Van Birgelen M. J. H. (2014). Value cocreation in service interactions: dimensions and antecedents. *Marketing Theory*.

[23] McColl-Kennedy J. R., Vargo S. L., Dagger T. S., Sweeney J., Van Kasteren Y. (2012). Health care customer value co-creation practice styles. *Journal of Service Research*.

[24] McColl-Kennedy J. R., Snyder H., Elg M. (2017). The changing role of the health care customer: review, synthesis and research agenda. *Journal of Service Management*.

[25] Zhaoquan J., Xiao X. (2015). Services innovation and value Co-creation under networked environment: a case study of ctrip. *Journal of Industrial Engineering and Engineering Management*.

[26] San-Martín H., Herrero Á. (2012). Influence of the user’s psychological factor on the online purchase intention in rural tourism: integrating innovativeness to the UTAUT framework. *Tourism Management*.

[27] Polo Peña A. I., Frías Jamilena D. M., Rodríguez Molina M. Á (2014). Value Co-creation via information and communications technology. *Service Industries Journal*.

[28] Poulis E., Poulis K., Doole L. (2013). ‘Information communication technology’ innovation in a non-high technology sector: achieving competitive advantage in the shipping industry. *Service Industries Journal*.

[29] Lan J., Ma Y., Zhu D., Mangalagiu D., Thornton T. F. (2017). Enabling value co-creation in the sharing economy: the case of mobike. *Sustainability*.

[30] Luu T. T. (2017). CSR and customer value co-creation behavior: the moderation mechanisms of servant leadership and relationship marketing orientation. *Journal of Business Ethics*.

[31] Vazquez-Casielles R., Iglesias V., Varela-Neira C. (2017). Co-creation and service recovery process communication: effects on satisfaction, repurchase intentions, and word of mouth). *Service Business*.

[32] Eisenhardt K. M. (1989). Building theories from case study research. *The Academy of Management Review*.

[33] Yin S. Q., Zhang J. L., Dou F. (2013). Standards and practice of scientific data monitoring in Europe-UKDA case study. *Library Journal*.

[34] Vargo S. L., Lusch R. F. (2004). Evolving to a new dominant logic for marketing. *Journal of Marketing*.

[35] Payne A. F., Storbacka K., Frow P. (2008). Managing the co-creation of value. *Journal of the Academy of Marketing Science*.

[36] Venkatesh V., Morris M. G., Davis G. B., Davis F. D. (2003). User acceptance of information technology: toward a unified view. *MIS Quarterly*.

[37] Fishbein M., Ajzen I. (1980). *Uncerstanding Attitudes and Predicting Social Behavior Prentice-Hall*.

[38] Mark P. Z., James M. O., Russell H. F. (1981). Self-perception and attitude-behavior consistency. *Personality and Social Psychology Bulletin*.

[39] Kan J., Tang Z. F., Sui H. (2016). Identification of key nodes of network public opinion based on Microblog information diffusion quality. *Information Science*.

[40] Yuan C., Hui L., Zhou W. H. (2015). Research on the application of big data in Taobao E-commerce model innovation. *Value Engineering*.

[41] Xueyan C., Duani F. F., Kuan F., Xian Z., Li S. M. (2014). Identification and classification of key nodes of public opinion in emergencies from the perspective of network forum. *Library And Information Service*.

[42] Taghizadeh S. K., Jayaraman K., Ismail I., Rahman S. A. (2016). Scale development and validation for DART model of value co-creation of innovation strategic process. *Journal of Business & Industrial Marketing*.

[43] Mazur J., Zaborek P. (2014). Validating dart model. *International Journal of Management and Economics*.

